# Role of senescence and mitotic catastrophe in cancer therapy

This article has been retracted.

**DOI:** 10.1186/1747-1028-5-4

**Published:** 2010-01-21

**Authors:** Richa Singh, Jasmine George, Yogeshwer Shukla

**Affiliations:** 1 Proteomics Laboratory, Indian Institute of Toxicology Research, (Council of Scientific & Industrial Research), PO Box 80, MG Marg, Lucknow-226001, India

## Abstract

Senescence and mitotic catastrophe (MC) are two distinct crucial non-apoptotic mechanisms, often triggered in cancer cells and tissues in response to anti-cancer drugs. Chemotherapeuticals and myriad other factors induce cell eradication via these routes. While senescence drives the cells to a state of quiescence, MC drives the cells towards death during the course of mitosis. The senescent phenotype distinguishes tumor cells that survived drug exposure but lost the ability to form colonies from those that recover and proliferate after treatment. Although senescent cells do not proliferate, they are metabolically active and may secrete proteins with potential tumor-promoting activities. The other anti-proliferative response of tumor cells is MC that is a form of cell death that results from abnormal mitosis and leads to the formation of interphase cells with multiple micronuclei. Different classes of cytotoxic agents induce MC, but the pathways of abnormal mitosis differ depending on the nature of the inducer and the status of cell-cycle checkpoints. In this review, we compare the two pathways and mention that they are activated to curb the growth of tumors. Altogether, we have highlighted the possibilities of the use of senescence targeting drugs, mitotic kinases and anti-mitotic agents in fabricating novel strategies in cancer control.

## Introduction

The incidence of cancer worldwide is on a rise, making it only second to coronary heart disease [1]. Unifying property of cancer includes six canonical characteristics: self sufficiency in growth signals, insensitivity to growth inhibitory signals (anti-growth), evasion of programmed cell death (apoptosis), unlimited proliferation of diseased cells, sustained angiogenesis, intrusion of adjacent cells and tissues and metastasis to distant niches in the body [2].

Genetic instability associated with telomere attrition or cell cycle checkpoint dysfunction is an early event in tumorigenesis. Telomeres are guanine rich tandem nucleotide repeats flanking the ends of chromosomes in all eukaryotic cells responsible for maintaining genetic integrity and implicated in aging (senescence) and cancer [3]. Cell cycle checkpoints or mitotic kinases (MKs) are the rigorous quality control steps of mitosis [4] that function in preserving the fidelity and integrity of DNA and allow mitosis to continue with accurately functioning DNA, spindle assembly, centrosome and kinetochore thus preventing cell death via mitotic catastrophe (MC). MC therefore, refers to the process when cells attempt to divide without proper repair of DNA damage due to faulty cell cycle checkpoint functioning consequently resulting in formation of giant, multinucleated cells with condensed chromosomes, distinguishing MC morphologically from other modes of cell deaths.

Abundant data amassed from several laboratories have provided innumerable instances to show that it is better to cure this dreadful disease at preventable stage by early diagnosis and consequent therapeutic intervention. Strategies for cancer treatment has generated significant interest in the recent past and therefore, the focus of research endeavors on understanding the mechanism of cell death pathways applicable in treatment of cancer which include not only apoptosis but necrosis, autophagy, MC and in context of cancer therapy, senescence has always been there [5].

This review will explore major highlights on the role of senescence and MC triggered in various cancers by chemotherapeutic intrusion and opens avenues for expanding research work by comparing the results obtained so far.

### Senescence: Terminal growth arrest in dividing cells

The term senescence is derived from the Latin word *senex*, meaning "old age" or "advanced in age". Senescence at the cellular level is a physiological program of cellular growth arrest that is triggered by the shortening of telomeres or by stress [6]. This permanent growth arrest is also considered a type of cell death in the context of cancer therapy by some researchers [7,8] and some consider it similar to the programmed cell death by 'apoptosis' [9]. Senescence can be broadly categorized into two classes: accelerated or stress induced premature senescence (SIPS) and replicative senescence (RS) and both are believed to be essential anti-carcinogenic programs in normal cells. Accelerated senescence occurs in response to the activation of Ras/Raf pathways [10] and by supra-physiological mitogenic signaling [11]. The phenomenon of RS was first described in the context of normal human cells explanted in culture that failed to divide beyond a finite number of fifty divisions [12] and it is a well-known defining property of euploid mammalian cells [13]. Telomere dynamics has been shown to be a critical component of both aging and cancer [14]. Telomeres, the highly repetitive DNA (TTAGGG sequence) which camouflages chromosome ends [15] prevent nucleolytic degradation, end-to-end fusion, irregular recombination, and other events that are normally lethal to a cell [15]. With each cell division a part of telomere gets eroded [16,17] and the chromosome being passed to the progeny gets the clipped off telomere.

Thus genetic integrity is gradually lost with telomeres progressively shortening after each division as a result of end-replication problems and hence, is a conspicuous feature in almost all dividing cells which do not express or maintain sufficient telomerase activity to maintain the telomeres. Telomerase reverse transcriptase (hTERT), whose amount is lessened after birth, functions by replenishing telomere by adding TTAGGG sequence at the 3'end of DNA. Telomerase activity is measured by TRAP assay or RT-PCR. Less frequently other alternative mechanism of telomere maintenance namely Alternative Lengthening of Telomeres (ALT) is opted [18]. Telomere dysfunction (short telomeres) has been associated with the initiation and progression of mouse and human intestinal neoplasia [19] and may also increase the risk of developing epithelial cancers by a process of breakage-fusion-bridge that leads to the formation of complex nonreciprocal translocations (a classical cytogenetic feature of human carcinoma) [20]. Blood relative telomere length was found to represent a strong independent prognostic indicator in patients with advanced breast cancer [21]. Similarly mean telomere length was statistically shorter in case patients with head and neck cancer as compared with control as measured with the southern blot and quantitative-fluorescent in situ hybridization assay [22]. Telomerase and p53 play critical roles in tumorigenesis and senescence. Senescent cells exhibit distinct morphology in culture. They are enlarged and flattened with increased granularity [23] exhibit SA-β-gal staining and a characteristic senescence associated heterochromatin foci (SAHF) formation [24] and comparatively less dense culture than a confluent young culture probably because they are more sensitive to cell-cell contact inhibition [12,13]. Even though they cannot divide under mitogenic stimulation yet they remain metabolically and synthetically active in *in vitro *conditions for several years [24] but can not resume cell growth after drug withdrawal. SA-β-gal, the most widely used surrogate marker with considerable specificity to senescent cells appears to reflect an increased lysosomal mass [23]. Another marker is clusterin/apolipopterin J, is a highly conserved ubiquitously expressed secreted glycoprotein has been implicated in many physiological processes, gets upregulated during stress induced premature senescence, *in vivo *aging, RS, in several age linked deformities, neuropathological disorders like Alzhiemers disease and dementia and has a direct relationship with human longevity [25]. Cellular senescence is a potent anti-cancer mechanism controlled by tumor suppressor genes, particularly p53 and pRb.

#### Role of p53

Telomere-induced senescence has been proved to be as effective as apoptosis in reducing cancer incidence and is mediated by the tumor suppressor gene, p53 [26]. Mutations in the p53 gene frequently appear in human tumors conferring aggressive oncogenic properties such as exacerbated malignant transformation and metastatic phenotype when over-expressed in p53-null cells. P53 gets activated upon genotoxic and non genotoxic stresses like oxidative damage and activates p21 and ultimately culminates the cell to senescence. Mice with a point mutation (p53(R172H)) in their endogenous p53 loci act as a model for the human Li-Fraumeni syndrome. Genetic alterations at chromosomes 3p, 6p, and 1lq were frequently found early in tumor development and showed additional allelic losses at chromosome arms 6q, 17p and 18q. Genes for telomerase suppression are presumably located on chromosomes 3, 4 and 6 [27].

P53 over expression has been directly associated with unfavorable clinico-pathologic factors such as advanced stage, histologic subtype, advanced patient age and nodal metastasis in endometrial carcinomas while bcl-2 expression was related with younger age, favorable grade and PR expression by tumor cells. Patient survival is however not related to the tested biomarkers [28]. In humans, TP53 codon 72 Arginine to Proline polymorphism was found to affect both cancer incidence and longevity as well [29]. The senescence-associated signature of p53 isoform expression (that is, elevated p53beta and reduced Delta133p53) was observed *in vivo *in colon adenomas with senescent phenotypes. The increased Delta133p53 and decreased p53beta isoform expression found in colon carcinoma may signal an escape from the senescence barrier during the progression from adenoma to carcinoma [30].

#### Other tumor suppressor genes

P107 is required for the initiation of accelerated cellular senescence in the absence of Rb and p130 may be required to prevent the onset of this phenomenon in un-stimulated prostate cancer cells lacking a functional Rb allele [31]. Cell cycle regulatory proteins are more sensitive to exogenous hormone treatment in postm-HBT (postmenopausal human breast tissue) than in pre-HBT (premenopausal human breast tissue) [32]. Olsson *et al *advocates that bfl-1 (tumor suppressor bcl-2 family member) contributes to chemo resistance and might be a therapeutic target in B-cell chronic lymphocytic leukaemia [33]. The activation of PI3K/Akt pathway is involved in the late-stage progression and metastasis of gastric cancer and attenuation of p-Akt by 2-ME suppresses metastasis [34]. Yet another tumor suppressor Promyelolytic leukemia (PML) regulates p53 acetylation in both RS as well as Ras induced accelerated senescence [35].

#### Senescence in cancer cells: In vitro studies

A large number of *in vitro *studies have been reported where a wide range of chemotherapeutical antidotes induce senescence like morphological changes and SA-β-gal expression in cancer cells activating the pathway of senescence. Research into the induction of cellular senescence as cancer therapy has however, been hindered by a lack of compounds that efficiently induce this response. To overcome this, Ewald *et al *(2009) by using dual Hoechst 33342 and SA-β gal staining identified library compounds that induce senescence in prostate cancer cells [36]. It is well acknowledged that telomerase and the maintenance of telomeres are key players in the ability of stem and cancer cells to bypass senescence and be immortal. Proliferation of telomerase (-) pre-malignant cells leads to telomere dysfunction and increased genomic instability suggesting one possible sequence of events leading to immortalization of breast epithelial cells during cancer progression [37]. The increased h-TERT expression may be a cellular response to genomic insults by various metal toxicants like arsenic that may also act as a tumor promoter in mammalian carcinogenesis as studied in blood cells by Mumford *et al *hTERT-specific T cells could contribute to the immunosurveillance of breast cancer suggests novel opportunities for both therapeutic and prophylactic vaccine strategies for cancer [38].

In one of the studies, using non-small lung adenocarcinoma A549 cells, it was shown that after treatment with DNA damaging anti-tumor drugs like caffeine, cells become permanently growth-arrested as a result of so-called drug-induced premature senescence (pseudo-senescence) or SIPS. Similarly, lowered efficacy of anti-cancer doxorubicin (due to dose dependent toxicity) against breast cancer cells can be increased when used in conjunction with siRNA inhibitor of telomerase [39]. Yet another study advocated the use ofGRN163L (novel telomerase template antagonist) in the treatment of breast cancer by augmenting the effects of paclitaxel [40]. Hence clearly proposing that inhibition of telomerase is a potential treatment strategy for inducing senescence. It has also been shown that caveolin-1 targets Mdm2/p53-mediated pathway and causes senescence in breast cancer cells [41]. Another study reported that bleomycin, a widely used anti-tumor agent, causes senescence of lung cancer cells by modulating the roles of caveolin-1, a protein abundant in lung fibroblasts and smooth muscle and endothelial cells [42].

A recent study showed that the activation of the p53-p21(Cip1/WAF1) pathway acts as a major mediator of cellular senescence induced by CKII inhibition in HCT116 colon carcinoma cells [43]. A senescence-inducing effect of doxorubicin on the same cells, in another study, had a dual effect-it stopped the proliferation of the majority of the cells and led to the appearance of proliferating aneuploid cells [44]. Likewise, while characterizing ashwagandha and its molecular mechanisms Wadhwa *et al *provided the first example that phytochemical(s) have both anti-cancer and anti senescent activities and pointed towards the molecular link between aging and cancer using normal human fibroblasts through decreased accumulation of molecular damage, down-regulation of the SA-β gal activity and the senescence marker protein, p21(WAF-1), protection against oxidative damage, and induction of proteasomal activity [45]. In one of the studies, by silencing BRCA1 expression at different levels through RNA interference technology in a series of partially transformed (HBL100) and tumorigenic (MCF7 and T47D) breast cancer cell lines, cell models were probed by clonogenic assay for their response to several DNA-damaging agents (mitomycin C, cisplatin, doxorubicin, and etoposide) commonly used in cancer therapy [46]. The increased sensitivity to these compounds displayed by BRCA1-defective cells was correlated to an increased fraction of growth-arrested, enlarged, multinucleated SA-β-galactosidase-positive senescent cells [46]. Melanocytic nevi frequently harbor oncogenic BRAF mutations and recently it was found that a subpopulation of melanocytes possess the ability to survive BRAF induced senescence, and suggest that p53 inactivation may promote malignant transformation of these cells [47] and thus have implications in skin cancer treatment. *In vitro *experiments with therapeutic nucleic acids successfully inhibited E6/E7 oncogene expression and caused induction of apoptosis and/or senescence in cervical carcinoma cells. A useful assay was described by Lau *et al *[48] to predict the response of the patient to a set of medicines without administering them by testing the susceptibility of a sample of cancer cells *in vitro *and comparing it to the standard regimen.

Apart from these, it has been observed that cells' passage number controls the appearance of senescence. Normal human diploid fibroblasts approach senescence near passage 64 through RNaseT2 expression, which however fails to induce senescence in SV40 immortalized cell lines [49]. Rat chondrocytes show the onset of senescence in the 4^th ^passage [50] while human rheumatoid arthritis fibroblast-like synoviocytes exhibit ageing at 10^th ^passage [51]. Stable clones derived from hTERT-expressing normal and G6PD-deficient fibroblasts have normal karyotypes, and display no sign of senescence beyond 145 and 105 passages, respectively, suggesting that ectopic expression of hTERT, in addition to telomere length maintenance by activating telomerase, also functions in regulating senescence induction [52]. Recently, a study explored the self-renewal potential of human breast stem cells and found that it gets exhausted within five *in vitro *passages of mammospheres, suggesting the need for further improvisation in culture conditions for their long-term maintenance [53].

#### Senescence in animal models: In vivo studies

Induction of senescence upon drug administration has been proposed as a possible anti-cancer treatment in various animal models. The finite proliferative potential of normal human cells leads to RS, which is a critical barrier to tumor progression *in vivo*. By studying embryonic fibroblast-derived cells with loss-of-senescence or H-RasV12/E1A-transformed phenotypes at different stages of oncogenic progression in nude mice, it was postulated that they may escape therapies aimed at metabolic inhibition of tumors with a fully developed Warburg phenotype [54]. β-carotene provides protection against O_3_-induced skin oxidative stress in female SKH-1 mice skin, which is consistent with a protective role for beta-carotene in the skin hence has implications in skin cancer and aging or senescence of skin [55]. A novel target of NESH-SH3 (TARSH), cellular senescence related gene in mouse embryonic fibroblasts may suppress tumor development in pulmonary tumorigenesis mouse model by causing an increase in SA-β-gal activity and this was attributed to p53-dependent p21^(Cip1) ^accumulation [56]. Pituitary tumor transforming gene deletion results in pituitary p21 induction and abrogates tumor development in Rb(+/-)Pttg(-/-) mice. Senescence was evidenced by increased p21 and SA-β-galactosidase. Aneuploid pituitary cell p21 may constrain pituitary tumor growth, thus accounting for the very low incidence of pituitary carcinomas [57]. Work by Efimova *et al *using p38-null mice skin carcinogenesis model strongly suggests a role for p38delta (key regulator in senescence, tumorigenesis, survival, inflammation etc) in promoting cell proliferation and tumor development in epidermis and may have therapeutic implication for skin cancer [58]. Three xenograft breast cancer mouse models, 2 of them with a TP53 mutation and one without it, were studied for their immediate response to high doses of epirubicin-cyclophosphamide. TP53 wild type stained positive for SA-β-galactosidase staining and also over expressed P21 but TP53 mutant did not succumb to senescence suggesting that treatment induced senescence is mediated via functional p53 in breast cancer [59]. More *in vivo *studies are however, needed to elucidate the role of senescence in cancer. Although these concepts are well supported in these models, translating them to clinical oncology remains a challenge.

#### Neosis - Achilles heel of cancer cells evading senescence

The physiological phenomenon of senescence serves as a lucrative pathway to annihilate deleterious cancer cells and tissues. This program of senescence is activated upon the administration of various anti-cancer regimens. Even though this is not a universal mechanism of curbing tumor cell growth, yet a considerable number of instances of *in vitro *as well as *in vivo *studies have been cited to decipher the metabolic pathway it targets and these studies have produced useful results that have enhanced and refined our knowledge about these pathways (Figure 1) and will be helpful in delineating new treatment strategies for curtailing cancer. Several studies [60,61], however provide compelling evidence that some cancer cells which are mitotically non-viable escape cell death, due to the accumulation of some genetic and epigenetic mutations and p53/pRB/p53^Ink4a^-dependent senescence checkpoint malfunctioning resulting in telomerase dysfunction [61,62] and finally evade cell death via continued progression through neosis. Such cells acquire so called' immortality' and to eliminate them, different strategies need to be designed. These cells multiply by a unique route called 'neosis' that facilitates in its progression and existence thereby evading the program of senescence. It has been described as a parasexual, somatic, reduction division in cancer [62]. Although neosis-like events have been reported in the literature sporadically for more than a century [63] under different names, they have been neglected due to the lack of appreciation of the significance of this process in cancer biology. Neosis may be a fundamental step in current concept of multi step carcinogenesis. Studying the behavior of individual neotic clones has revealed the significance of their central role in cancer [64]. Non-synchronous occurrence of secondary/tertiary-neosis (Figure 2) creates the illusion of the existence of cancer stem cells and the 'mirage' of immortality of cancer cells.

**Figure 1:** **Genes involved in senescence**.

**Figure 2:** **Prerequisites for the onset of neosis and step-wise depiction of primary neosis (P/neosis) and secondary and tertiary neosis (S/T neosis)**. When a normal diploid cell accumulates genetic mutation owing to exposure, either dies following apoptosis or necrosis or may enter mitotic crisis and after repair again re-enters cell cycle or may become tetraploid after few hours or become polyploidy and succumb to senescence or may circumvent senescence and divide by neosis. Neosis of non-viable NMCs may give rise to genetically viable daughter cells 'Raju cells' by P/neosis and further divide and re-divide by S/T neosis. The number of progenies may vary from one to infinite and differ from NMCs and other daughter cells unlike conventional mode of division, mitosis. Number of surviving progenies depends on the 'survival of the fittest'.

Some of the genetic and epigenetic alterations become the achilles heel of the mutated tumors that bypass the effect of certain classes of anti-cancer agents. That is, patients whose tumors carry such defects can be stratified for respective therapy rendering some classic DNA damaging agents called neosicides into "targeted therapies." Development of novel strategies to improve current status of cancer therapy will require identification and exploitation of yet unrecognized differences between normal and tumor cells with respect to propagation, evolution and development of resistance to conventional treatments [65]. The discovery of neosis has identified novel cellular targets, against which one can identify novel neosis-specific molecular targets in order to design anti-neotic agents or neosicides that will be more specific in their action and do less harm to non diseased cells. A judicial combination of senescent drugs with efficient neosicides could further improve the status of cancer control.

### MC and role of MKs in cancer

According to the tenets of cancer biology, tumor cells arise after about 13 mitotic divisions of the initiated cell [66]. MKs, are rigorous quality control steps of mitosis and function in preserving the fidelity and integrity of DNA and allow mitosis to continue only with accurately functioning DNA, spindle assembly, centrosome and kinetochore thus preventing MC [67]. Malfunctioning of MKs are intimately involved in the development of errors in a vast majority of solid tumors and hematological malignancies. MC is an event in which a cell is destroyed during mitosis. This is believed to be caused through apoptosis as a result of an attempt at aberrant chromosome segregation early in mitosis, or as a result of DNA damage later, during the metaphase/anaphase transition. Cells which fail to go through a MC after mitotic failures are likely to create aneuploid cells when they later reproduce, posing a risk of oncogenesis, potentially leading to cancer [67]. Hence MC is also in the league of processes which participate in prevention of cancer. MC which has been described as 'Death through a tragedy' [68] is stimulated by ionizing radiations (IR), chemotherapeutic drugs or hyperthermia and is caused by malfunctioning of cell cycle checkpoints and MKs. The normal choreography of the events in the mitotic cell cycle gets disturbed and aneuploidy follows. An aneuploid cell can be hyperaneuploid and may contribute to tumorigenesis by an enhanced expression of oncogenes or may be hypo-aneuploid and be liable for tumorigenesis by a loss of heterozygosity of various tumor suppressor genes [69].

MC shares several biochemical hallmarks of apoptosis, in particular mitochondrial membrane permeabilization and caspase activation [70] but is proposed to be fundamentally different from apoptosis [71]. Both senescence and MC are important pathways that cause cell annihilation upon chemotherapeutic intervention. The mechanism and morphology of the deceased cells is however different in both the cases. A tabular representation of the differences between MC and senescence is given in Table 1.

**Table 1:** Comparison between senescence and mitotic catastrophe

Characteristics	Mitotic catastrophe	Senescence
Definition	Synonymous with 'Terminal proliferation arrest' may proceed with apoptosis or necrosis depending on molecular profile of the cell	Synonymous with 'Terminal growth arrest' Cell death in context of cancer
Biomarker	Multinucleated giant cells, no specific *in vitro *and *in vivo *assay available	SA-β galactosidase expression, detected by X-gal staining
Morphology	Aneuploidy, disrupted DNA index, micronuclei formation, nuclear envelope lacking, nuclear fragmentation and uncondensed chromatin	Flattened enlarged cells, granular cytoplasm, exhibit SAHF formation
Genotype implicated in carcinogenesis	Accelerated by G1, G2 and prophase checkpoint proteins (ATM, ATR, p53, Chk2, Cdc25A, Cdc25B, Plk1 & 3)	Accelerated by telomere attrition, ras mutations, inhibited by ALT or p53
Inducing agents	Hyperthermia, IR, anti-cancer drugs interfering with DNA or microtubule assembly	Spontaneous as a result of cumulative divisions or challenged by oncogenic stimulus

Genetic checkpoint defects lead to syndromes that demonstrate chromosomal instability, increased sensitivity to genotoxic stress and consequently cancer predisposition. The detection of persistent MK over-expression, particularly the Aurora kinase family, and centrosome amplification in precursor/pre-malignant stages, strongly correlate these molecular changes in precipitating the aneuploidy seen in many human neoplasms [72]. The sustained over-expression and activity of various members of the MK families, including Aurora kinases (A, B, C), Polo-like (Plk1-4), and Nek (NIMA1-11) in diverse human tumors strongly indicate that these entities are closely involved in the development of errors in centrosome duplication, chromosome segregation, and cytokinesis.

#### MKs families

The focus of this section is on the different MKs families. These kinases are modulated by de-novo synthesis, stability factors, phosphorylation, and ubiquitin-dependent proteolysis. They, in turn, phosphorylate innumerable centrosomal/mitotic protein substrates, and have the ability to behave as oncogenes (i.e. Aurora-A, Plk-1), providing a compelling link between errors in mitosis and oncogenic processes [73]. Additionally, dysregulation of MKs have been linked with improper cell cycle progression both *in vitro *and in vivo. Without getting into the basics of MKs, the main pre-clinical and clinical studies concerning MK inhibitors currently under investigation are reported and important considerations for their future development are discussed. Here is given a representation of kinases in different phases of cell cycle (Additional File 1: Table S1).

#### Cyclin dependent kinases 1 (Cdk1)

Cdk1 is vital participant in the mitotic cell cycle. Mitosis begins and ends with the activity of cdk1 with binding partner cyclin B1. First studied in fission yeast (*Saccharomyces cerevesiae*), Nurse [74] identified a gene that controlled mitosis and named it cdk1 or cdc2. Studies have revealed that functional p53 protein may enhance the anti-cancer activity of roscovitine (known cdk1 inhibitor) that could be beneficial for anti-cancer therapy [75]. Tumorigenecity mediated by p53 loss does not require either Cdk2 or Cdk4, which necessitates consideration of the use of broad spectrum cell cycle inhibitors as a means of effective anti-Cdk cancer therapy [76]. Gartner *et al *have reported for the first time reported an association of cyclins and Cdks with the microtubule network by immunoelectron microscopy and immuno-biochemical methods. Cyclins D, E, A and B as well as Cdks 1, 2 and 4 were also found to be associated and exhibit kinase activity towards the microtubule-associated protein tau [77]. Bailet *et al *[78] have highlighted a new role for spleen tyrosine kinase (Syk) in regulating cellular senescence and identify Syk-mediated senescence as a novel tumor suppressor pathway, the inactivation of which may contribute to melanoma tumorigenicity. Study by Buchanan *et al *[79] on murine adenocarcinoma mammary cells provided new clues regarding the mechanism involved in the modulation of mammary tumor cell growth and survival induced by glypican-3. Gene expression profiling has generated hypotheses that led to an increase in our knowledge of the cellular effects of seliciclib (cdk inhibitor) and could provide potential pharmacodynamic or response biomarkers for use in animal models and clinical trials [80]. Another Cdk inhibitor SU9516 is over expressed in HCT116 cells by the knockout of the p21^WAF1/CIP1 ^gene which suppresses thymidylate synthase and enhances chemosensitivity to 5-Flurouracil [81].

#### Check point kinases 1 (Chk1) and 2 (Chk2)

Chk1 and Chk2 are effector kinases in the cellular DNA damage response and impairment of their function is closely related to tumorigenesis. If DNA damage is detected after S and before G2/M transition, ATM/ATR is activated and phosphorylation of Chk1 and Chk2 occurs [82] leading to cell death during mitosis or MC. Experiments have demonstrated that there are alternate mechanisms for activating ATM that are both stress-specific and independent of the presence of DNA breaks [83]. The activation of the ATR-Chk1 pathway in response to bifunctional DNA alkylator 1,3-bis(2-chloroethyl)-1-nitrosourea (BCNU) treatment and the dependency of this response on the DNA mismatch repair capacity were investigated. Chk1 was found to be phosphorylated at serine 345 and exhibited increased kinase activity. Si-RNA knockdown of ATR also reduced Chk1 phosphorylation following exposure to BCNU. However, knockdown of ATM had no effect on the observed Chk1 phosphorylation, suggesting that ATR was primarily responsible for Chk1 activation [84].

#### Polo like kinases (Plk)

A family of serine/threonine kinases also designated as tubulin-associated proteins actively participate during mitosis and comprises four distinct members: Plk1 (Plk), Plk2 (Snk), Plk3 (Prk or Fnk) and Plk4 (Sak) [85] each carrying out a multitude of distinct roles. Plk1 is the most extensively characterized among the family members, suggesting that the polo box domain of it can provide an additional structural basis for discovery of new anti-cancer drugs. It was also found out that Plk1 is required for chromosomal DNA replication under stressful conditions [86] and Plk3 is more potent in inhibiting cell proliferation and inducing apoptosis [87].

Plk1 gene expression is tightly regulated with mRNA increase beginning in S phase and peak mRNA levels detected at G2-M transitions and through mitosis [88]. RNA-interference -mediated depletion of Plk1 to determine its potential for sensitizing pancreatic tumor cells to gemcitabine showed that small interfering RNA-mediated knockdown of Plk1 caused cell cycle arrest at G2/M and the reduction of cellular proliferation and decreased cell viability and increased cellular apoptosis [89]. Transcription of Plk1 is inhibited along with other G2/M specific genes like cyclin B1, cyclin B2 and cdc25B by inhibition of Nuclear Factor kappa B at G2-M phases [90]. Studies define and illuminate a late mitotic function of Plk1 that it is obligatory in the positioning and recruitment of Rho guanine nucleotide exchange factor (RhoGEF) Ect2 to the central spindle and abolishing RhoA GTPase localization to the equatorial cortex, and suppressing cleavage furrow formation and cell division [91]. Increased *plk-1 *gene and protein perhaps play a key role in abnormal proliferation of acute leukemia cells and correlate with the malignancy of leukemia [92] prostate carcinoma, [93] and gastric carcinoma [94]. Snk/Plk2 is transcriptionally down-regulated in B-cell neoplasms [95] and consequently provides a potential mechanistic basis underlying the strong selective pressure for abrogation of Plk2 function in B-cell neoplasia. Plk3 has been shown to catalyse the priming of Cdc25A by phosphorylated glycogen synthase kinase-3β (GSK-3β) and observations indicate that GSK-3β inactivation may account for Cdc25A overproduction in a subset of human tumors [96]. LFM-A13 (alpha-cyano-beta-hydroxy-beta-methyl-N-(2,5-dibromophenyl)propenamide) has recently been identified as an inhibitor of Plks and markedly enhances the anti-cancer activity of paclitaxel [97] with anti-proliferative activity against human breast cancer [98].

#### Aurora kinases

Aurora kinases namely, Aurora A(Aurora 2), Aurora B(Aurora 1) and Aurora C(Aurora 3) are serine/threonine kinases also known as tubulin-associated proteins [99] which are expressed only in actively dividing cells and their increase is a factor of bad prognosis in cancer. Side effects, dosing and tolerability of inhibitors have been discussed in great length by Pinel *et al *[100] and enzymatic characterization of GSK1070916, a potent and selective Aurora-B/Aurora-C inhibitor was done and compared with other Aurora inhibitors AZD1152 and VX-680 [101], GSK1070916 was found to exert a more prevailing inhibitory effect due to a slow rate of dissociation from the Aurora-B & C enzymes. Detailed kinetic analyses of two isogenic cell lines differing in p53 function and have been compared with the effects of ZM447439 and VE-465 to describe several mechanisms explaining how cells may evade killing by Aurora kinase inhibitors [102]. It has been proposed that perikinetochoric rings of MCAK and Aurora-B define a novel transient centromere domain at least in mouse chromosomes during meiosis and also its functions have been illustrated by Parra *et al *[103].

#### Bub related kinases (Bub family)

The Bub family of kinases constitutes members that are concerned with spindle assembly functioning and APC/C regulation. In one of the studies p53 was sustained to express in K562 leukemic cells after being infected by recombinant adenoviruses carrying the wt-p53 gene and it was shown that wt-p53 can suppress excessive replication of centrosomes and may contribute to the upregulation of Gadd45a and BubR1 protein expression as well as the downregulation of Aurora A protein expression [104]. A novel study reports that Ajuba, a microtubule-associated protein collaborates with Aurora B and BubR1 at the metaphase-anaphase transition and ensures proper chromosome segregation[105].

#### Never in mitosis A- Related kinase (NIMA, Nek, Nrk)

The Nek or Nrk related kinase family are essential MKs first described in the filamentous fungus Aspergillus nidulans [106] containing 11 members (Nek1, 2, 3, 6, 7, 8, 9, and 11 are prominent) [107]. Nek1 is involved early in the DNA damage sensing/repair pathway after IR and G(1)-S-phase checkpoint control can be rescued by ectopically over-expressing wild-type Nek1. Moreover, in cells without functional Nek1, DNA is not repaired properly, double-stranded DNA breaks persist long after low dose IR, and excessive numbers of chromosome breaks are observed [108]. Recently, studies have explicated that ciliary localization of Nek8 in a subset of ureteric-bud-derived kidney tubules is essential for maintaining the integrity of those tubules in the mammalian kidney [109].

#### MKs and their role in cancer control- In a nutshell

As current cancer therapies are still in their infancy and are not able to fulfill the expectations of cancer control, strategies targeting mitotic regulators could be a potentially pragmatic option, which may improve the therapeutic index when used either alone or in combination with current anti-cancer antidotes. The uniqueness of MKs lies in the fact that they are expressed in actively duplicating cells and not in differentiated cells further make it important targets against cancer cells. Targeting MKs would aid us in understanding the mechanism of chemo-resistance. The research efforts to examine the role of MKs and mitotic signaling pathways are, however, in its beginning. By presenting an overview of regulation of MKs in this review, we open promising avenues in designing novel therapeutic approaches in curbing cancer. Simultaneously, we also present the rationale for these kinases as an anti-cancer target. Hence, more concern needs to be laid on *in vivo *work to understand the role of MKs and their utility as targets before we can actually embark on translational studies in human.

## Conclusions and future connotations

Cancer is a global health problem and various treatment strategies are premeditated for curbing this deadly biomedical manifestation. Cells continuously encounter DNA damage caused either by damaging agents, including oxygen radicals and DNA replication errors caused by stalled replication forks, or by extracellular environments such as ultraviolet or IR. The cellular response to radiation or chemicals is complex and may lead to different biological outcomes. Senescence, MC, necrosis, apoptosis and autophagy are such mechanisms out of which the two former mechanisms have been discussed in this review.

The physiological phenomenon of senescence is stimulated by ras/raf activity, telomere attrition and p53. Cellular senescence is a persistently growth-arrested phenotype in normal and transformed cells which may be beneficial when used to target the proliferation of tumor cells or during organogenesis or wound healing. It is well known that cancer risk rises exponentially with age fuelled by somatic mutations. Senescence leads to altered expression of genes (cell division control, cell structure and metabolism) and imparts resistance to cells towards apoptosis apart from actively secreting inflammatory cytokines, proteinases and growth factors. Keeping all these aspects about this mechanism in mind, we can design novel treatment tactics in curbing cancer. The discovery of neosis has identified novel cellular targets, against which one can identify novel neosis-specific molecular targets in order to design anti-neotic agents or neosicides that will be effective against many tumor types and theoretically be expected to have a prophylactic action against multiple primary cancer growths.

Discussing the regulation of MKs, we open promising avenues in designing novel biomarkers for novel unexplored targets and present the rationale for these kinases as an anti-cancer target. More *in vivo *work needs to be undertaken to understand the role of MKs and their prospective as cellular targets before translational studies can be performed in humans. Several key works using clinical samples strongly suggest that point mutations of the checkpoint genes contribute to malignant transformation and genetic instability in cancer cells. However, the exact role of DNA damage checkpoints in the prevention of human carcinogenesis should be re-evaluated. The spindle checkpoint inhibits the ubiquitin ligase activity of the anaphase-promoting complex or cyclosome (APC/C), which is essential for mitotic progression, until spindles are properly attached to all kinetochores, and thus prevents precocious chromosome segregation. Because in a large proportion of tumors, cell cycle checkpoints are compromised and apoptotic pathways frequently suppressed, tumor cells preferentially execute this mitotic mode of cell death after treatment with DNA damaging regimens. A judicial combination of anti-neosicides and anti-mitotic agent may increase the therapeutic ratio under clinical settings. Moreover, results of recent important research work on senescence and MC can lay foundation of other experiments targeting different cancers for testing efficacy of already tested drugs and on some cancers for different drugs sharing similarities in chemical and physical properties with known drugs.

## Conflict of interests

The authors declare that they have no competing interests.

## Authors' contributions

RS composed the original manuscript. JG made extensive revisions and participated in manuscript preparation. YS edited and finalized the final manuscript. All authors read and approved the final manuscript.

## Supplementary Material

Additional file 1 **Table S1**. Roles of various kinases and substrates during different cell cycle phases Click here for file
